The article "The Method for Identifying Employees' Emotions in Adverse States Incorporating PSO-kNN Algorithm and Multiple Physiological Parameters" was published in 2022. Journal: Comput Intell Neurosci.

# The Method for Identifying Employees' Emotions in Adverse States Incorporating PSO-kNN Algorithm and Multiple Physiological Parameters

**DOI:** 10.1155/2022/4371162

**Published:** 2022-04-23

**Authors:** Jiaonan Han

**Affiliations:** Human Resources Business Consulting Department, Kunlun Digital Technology Co. Ltd., Beijing 100007, China

## Abstract

It is well known that we, as human beings, are prone to a variety of undesirable emotions such as excitement, boredom, and fear, all of which are induced by varying degrees of negative states. In this paper, we designed an emotion-evoking experiment to induce calm, excited, bored, and fearful emotions, as well as low, moderate, and high levels of tension. Based on the six physiological signals such as heart rate and respiration rate of the subjects in these emotion states, feature extraction was performed after removing the baseline preprocessing, combined with particle swarm optimisation algorithm for feature selection, and the k-nearest neighbour algorithm was used to classify the different emotion and tension levels in the undesirable states. By comparing the results of several sets of experiments, we found that with baseline removal and particle swarm feature selection optimisation, our experimental results using k-nearest neighbour classification showed a significant improvement in recognition accuracy compared to the traditional k-nearest neighbour algorithm, which indicates that the proposed method has better recognition results.

## 1. Introduction

Emotions are a combination of states that arise when a person is exposed to external stimuli. A good emotional state is conducive to maintaining physical and mental health, while chronic bad moods can have a great impact on a person's mental health and physical health. For example, prolonged bad moods can easily lead to depression, which affects one's social functioning and interpersonal interactions and can even be life-threatening [1]. For people with cardiovascular diseases, extreme emotions such as anger and anxiety can increase the risk of morbidity. Anger generated by drivers during driving can easily trigger road rage, which can seriously affect the life safety of drivers and other traffic participants, etc. In summary, emotions have a significant impact on all aspects of human life, so it is particularly important to identify them accurately.

At the present stage, the way of emotion recognition is mainly divided into two aspects; one is recognition through nonphysiological signals such as human facial expression, voice tone, and body posture [2], because these nonphysiological signals can be artificially controlled by means of camouflage and other means, resulting in sometimes not being able to obtain the real signal that can represent the emotion, thus not being able to accurately identify the real emotional state. On the other hand, physiological signals such as EEG signals, electro-ocular signals, ECG signals, EMG signals, and skin current responses can be used for emotion recognition [3, 4]. Emotion recognition based on physiological signals can obtain more objective and realistic results, which is also more conducive to practical applications [5].

The article "The Method for Identifying Employees' Emotions in Adverse States Incorporating PSO-kNN Algorithm and Multiple Physiological Parameters" was published in 2022. Journal: Comput Intell Neurosci.

An adverse state in the article is a combination of physical and mental reflections when people find that something real or imagined is beyond their expectations [6]. Chronic stress can lead to an increased susceptibility to illness, which can induce a variety of diseases [7]. In terms of emotions themselves, there is an important correlation between them and dysphoric states. Often, people wear black in bad states with a variety of complex emotions, of which excitement, fear, and boredom are more common [8]. In contrast, emotions are expressed differently as a mental feeling and state, which often requires the use of language, tone of voice, facial expressions, behavioural gestures, breathing, and other media [9]. Physiological signals are more objective and realistic in reflecting people's emotional state and psychological feelings at the time [10].

The theory of “affective computing,” which reflects specific emotions through changes in physiological signals, was first proposed by Professor Pi card [11] at the MIT, who suggested the feasibility of extracting features from physiological signals for emotion recognition [12]. Nasoz et al. [13] from the University of Central Florida, USA, used *k*-nearest neighbour (kNN), Discriminant Function Analysis (DFA), and Marquardt back propagation (MBP). Kim et al. of Yonsei University, Korea [14], used the Support Vector Machine (SVM) algorithm; the Institute for Computational Science at the University of Augsburg, Germany, focused on comparing the recognition effects of combining different feature selection methods and classifiers [15]. The research on emotion computing in China started late, among which Guangyuan Liu's team from Southwest Jiaotong University conducted a comparative study on the effect of emotion recognition on emotion data samples from Augsburg University using a combination of various feature extraction and selection methods and classifiers [16].

Zhai et al. [17] used the SVM algorithm, and Setz et al. [18] carried out the classification using DFA and SVM algorithms. At present, there are relatively few studies at home and abroad on affective computing in adverse states, especially for different stress levels. The particle swarm optimisation (PSO) algorithm is combined with the kNN algorithm to investigate the identification of emotional experiences under adverse states based on multiple physiological signal parameters. Based on the removal of baseline emotions, the PSO algorithm optimises the selection of multiple features of multiple physiological signals and then uses kNN for classification to obtain better recognition results. The highest recognition rate reaches over 80%, which improves the correct rate of the traditional method of recognising emotional states with multiple physiological signals [19] and provides a way to explore the relationship between emotions in adverse states, and this provides a basis for exploring the relationship between emotions and multiple physiological signals in adverse states.

The article "The Method for Identifying Employees' Emotions in Adverse States Incorporating PSO-kNN Algorithm and Multiple Physiological Parameters" was published in 2022. Journal: Comput Intell Neurosci.

## 2. Research Methods for Identifying Emotions in the Adverse States

This study firstly designed different emotion and tension level evoking experiments under adverse states and collected six physiological signal parameters such as heart rate, respiration rate, skin impedance, blood oxygen saturation, pulse rate, and blood pressure under specific emotional states of multiple subjects in real time. Through preprocessing and feature extraction of these physiological data, combined with the results of the experimental subjective experience questionnaire, the PSO-kNN algorithm was used to select and classify the features of the experimental sample data and finally to establish the emotion recognition model under the adverse state [20].

### 2.1. Particle Swarm Algorithms

The algorithm is conceptually simple, easy to implement, and fast to converge, has few parameter settings, and is little affected by changes in feature dimensions, making it an efficient search and optimisation algorithm [21]. Therefore, this paper uses the particle swarm algorithm for feature optimisation selection of physiological features.

Assuming that the total number of features is *D* and there are *m* individuals in the population, the velocity of the ith particle is *V*_*i*_=(*v*_*i*1_, *v*_*i*2_, *v*_*i*3_,…,*v*_*i*  *D*_)^*T*^, its position is *X*_*i*_=(*x*_*i*1_,  *x*_*i*2_,  *x*_*i*3_,   ⋯ , *x*_*i*  *D*_)^*T*^, and the value of the position is a solution. By comparing the fitness values, the optimal position experienced by the current *i*th particle can be obtained as Pbest_*i*_=(pbest_*i*1_, pbest_*i*2_, pbest_*i*3_, ⋯,pbesti_*D*_)^*T*^ and by comparing all particles, the optimal position of the whole population can be obtained as Gbest=(gbest_1_, gbest_2_, gbest_3_, ⋯,gbest_*D*_)^*T*^.

(1) $$\begin{array}{c} V_{i}^{n+1}=w\times V_{i}^{n}+C_{1}\times {\text{ rand}}_{1}\left(\;\right)\times \left({\text{Pbest}}_{i}-X_{i}^{n}\right)+C_{2}\times {\text{rand}}_{2}\left(\;\right)\times \left(\text{Gbest}-X_{i}^{n}\right), \end{array}$$

(2) $$\begin{array}{c} X_{i}^{n+1}=X_{i}^{n}+V_{i}^{n}, \end{array}$$

where *w* is the inertia weight factor, usually with values 0.4 to 0.9. *C*_1_ and *C*_2_ are the learning factors, and usually, *C*_1_=*C*_2_=2. rand_1_() and rand_2_() are the random vectors between 0 and 1. A too-large inertia weight can increase the flight speed of the particles, which is conducive to jumping out of the local extremes, which makes the particles search locally. According to (3), let the inertia weight linearly decrease with the number for weight adjustment, faster to achieve convergence of the algorithm.

(3) $$\begin{array}{c} w\left(t\right)=w_{\max}-\left(w_{\max}-w_{\min}\right)\times \frac{T}{T_{\max}},T=1,2,..,T_{\max}, \end{array}$$

where *w*_max_ is the maximum value of inertia weight, *w*_min_ is the minimum value of inertia weight, *T*_max_ is the maximum number of iterations, and *T* is the current number of iterations. The initial values of the parameters in this paper are set using the inertia weight method [22], where *w* will be initialized to a constant 0.729 and *C*_1_=*C*_2_=1.494. To prevent particles from flying out of the search space, *V*_*i*_ ∈ [−*V*_max_, *V*_max_] is generally taken; *V*_max_ will be too large to fly away from the best solution, and too small value will fall into a local optimum.

The article "The Method for Identifying Employees' Emotions in Adverse States Incorporating PSO-kNN Algorithm and Multiple Physiological Parameters" was published in 2022. Journal: Comput Intell Neurosci.

### 2.2. The k-Nearest Neighbour Algorithm

The kNN algorithm is a well-established and simple classification algorithm that makes full use of the physiological features of the entire emotion sample. The kNN algorithm, a commonly used classification algorithm, works on the principle that a sample is defined as belonging to a class if the vast majority of its sample points in the feature space belong to that class within a neighbourhood [23]. kNN algorithm is an algorithm in which the selected neighbours are all objects of the training set that have been correctly classified. The nearest neighbour parameter is set to 1 in this paper.

### 2.3. PSO-kNN Algorithm

In the PSO-kNN algorithm [24], a particle is considered to have a higher fitness value when the number of features it produces is smaller and its classification accuracy is higher. The fitness function for evaluating each particle is *f*(*x*). The larger the *f*(*x*) is, the better the fitness is, and the fitness function can be defined as follows:

(4) $$\begin{array}{c} \text{ fitness}=\frac{1}{\text{ RMSE}\times \text{Factor}+\text{Features}}, \end{array}$$

where  RMSE is the root mean square error, Features is the number of subsets of sample features, and Factor is the balance factor. We have the following steps:

 
*Step 1*. Design particles, represented by a binary bit string, with each binary bit corresponding to a feature in the physiological signal feature set, where a 1 in the bit indicates that the corresponding feature is in the selected feature subset and a 0 in the bit indicates that the corresponding feature is not in the selected feature subset [25].
 
*Step 2*. Initialize the particle swarm, i.e., set the *X*_*i*_ and initial velocity *V*_*i*_ of each particle at random.
 
*Step 3*. Learn and train with the kNN algorithm, and calculate the particle fitness according to equation (4).
 
*Step 4*. For each particle, compare the fitness function value *f*(*x*_*i*_) with its own optimal value *f*(pbesti), and if *f*(*x*_*i*_) < *f*(pbesti), replace the previous round's optimal value with the fitness value and replace the previous round's particle with the new one.
 
*Step 5*. Compare the best-fit value *f*(*x*_*i*_) of each particle with the best-fit value *f*(pbesti) of all particles. If *f*(*x*_*i*_) < *f*(pbesti), replace the original global best-fit value with the best-fit value of that particle, while saving the particle.
 
*Step 6*. The particles according to model equations (1) and (2) of PSO produce a new population *X*_*i*+1_ with the following velocity adjustment rules: when *v*_*i*_ > *V*_max_, *v*_*i*_=*V*_max_; when *v*_*i*_ ≤ −*V*_max_, *v*_*i*_=−*V*_max_.
 
*Step 7*. Update the inertia factor *ω*.
 
*Step 8*. Update the binary bits of the particle.
 
*Step 9*. Check the end condition. If it is satisfied, the search ends and the current optimal feature subset and classification accuracy are returned; otherwise, the number of iterations is increased so that iteration *T*=*T*+1 is reached and the search ends at the maximum number of iterations *T*_max_ or the evaluation value is less than the given accuracy.

The article "The Method for Identifying Employees' Emotions in Adverse States Incorporating PSO-kNN Algorithm and Multiple Physiological Parameters" was published in 2022. Journal: Comput Intell Neurosci.

## 3. Emotion-Evoking Experiments

### 3.1. Experimental Materials

The International Affective Picture System (IAPS) [26] from the NIMH Emotion and Attention Research Center at the University of Florida was used as the main material for the different emotion elicitation experiments in adverse states. These selected images were assessed for validity and arousal by a large number of subjects in different emotion elicitation experiments to determine the reliability of this approach. In this process, the validity and arousal are determined by the size of the defined data, where smaller numbers indicate lower validity and arousal and larger numbers indicate higher validity and arousal. Elicitation experiments for different levels of tension in the dysphoric state were elicited using different digit addition and subtraction mental arithmetic tasks. The efficacy values and arousal levels for the four IAPS emotionally arousing picture materials are given in Table 1.

A visual comparison of the effect of these four emotionally evocative picture material values and arousal levels is shown in Figure 1.

### 3.2. Experimental Subjects

There were 14 subjects (8 males and 6 females) from Shanghai Jiaotong University, aged 22 to 27 years old. They were physically and mentally healthy, had normal vision and hearing, had no previous history of psychiatric or neurological disorders, and had participated voluntarily in the experiment. They were not involved in strenuous exercise within 4 hours prior to the experiment and did not use any drugs within one week prior to the experiment. Before the start of the experiment [27], each subject was made fully aware of the purpose and procedure of the experiment and was tested with a stress-tolerance questionnaire, and all had a certain level of stress tolerance. The whole experiment was conducted in strict compliance with the Declaration of Helsinki.

### 3.3. Experimental Equipment

A high-performance computer system (Intel(R) CoreTM i5-2310 CPU @2.90 GHz, 4 GB DDR3RAM, Lenovo, China; 17-inch professional display, 300 *c*  *d*/*m*^2^, resolution 1280 × 768, vertical refresh rate 75 Hz) was used for the presentation of the emotionally evoked material. The screen for the presentation of pictures and mental arithmetic questions is approximately 50 cm away from the subject. Physiological signals are detected and recorded based on a portable multiphysiological parameter acquisition device developed by the laboratory, which can acquire a variety of physiological signal parameters such as ECG, heart rate, respiration rate, skin impedance, oxygen saturation, pulse rate, and blood pressure. The heart rate can be monitored from 30 bpm to 240 bpm with an error of≤2%, respiratory rate≤5%, skin impedance≤3%, blood oxygen≤2%, pulse rate ≤3%, and blood pressure within ±1.3 kPa (10 mmHg).

### 3.4. Experimental Procedure

**Experiment 1 .**

Firstly, in an emotion-evoking experiment with different visual stimuli, each of the ten emotion-evoking pictures of the same type was presented in sequence for 12 s. The whole process was completed in 2 min. The subjects took 2 min to calm down after each slide show and assessed the emotion elicited by the pictures. Before the start of the experiment, each participant was given a set of pretests to familiarise them with the process and the experimental environment. The preexperiment images were also taken from the IAPS.

The article "The Method for Identifying Employees' Emotions in Adverse States Incorporating PSO-kNN Algorithm and Multiple Physiological Parameters" was published in 2022. Journal: Comput Intell Neurosci.

**Experiment 2 .**

For the elicitation of tension in different difficulty tasks, elicitation of tension in adverse states by giving two-digit, three-digit, and four-digit addition and subtraction mental arithmetic tasks with different levels of difficulty was done [28]. Each question was presented for 5 s, for a total of 125 s. Subjects were told to complete all questions as correctly as possible within the time limit, with an additional bonus if they obtained 95% or more score. Subjects were given a 2 min break between each set of questions to allow for emotional recovery. After the three sets of mental arithmetic tasks were completed [29], subjects were asked to give a subjective assessment of the level of tension induced by the three sets of tasks. Before the start of the experiment, a pretest was also conducted to familiarise the subjects with the procedure.

### 3.5. Experimental Data Processing

A total of 98 samples of physiological signals were obtained from 14 subjects through the tension elicitation experiment under different emotions and different difficulty tasks. Based on the subjects' subjective questionnaires [30], a total of 89 valid physiological signals were selected. Among them, 14 were calm, 10 were fearful, 12 were excited, 11 were bored, 14 were low tension, 14 were moderate tension, and 14 were high tension. In order to eliminate the differences in physiological data between subjects, the baseline physiological data of each subject in a calm emotional state were subtracted from the sample data obtained under fear, excitement, boredom, low tension, moderate tension, and high tension to obtain the baseline physiological sample data, i.e., 33 samples of the three types of emotions and 42 samples of the three tension levels. After completing the preprocessing of the data, feature extraction was performed on the various types of physiological signal data samples according to Table 2 and 33 features were finally obtained.

The specific distribution structure of the features extracted from the six physiological signals is illustrated in Figure 2.

## 4. Experimental Results and Analysis

In the emotion elicitation experiments of the article, the emotion recognition algorithm performed on the basis of adverse states with multiple physiological signals was implemented on Matlab 2019a. For the 33 samples in the target, 21 of them were randomly selected as the training set and the remaining 12 samples were used to test the experimental results. In order to fully validate the experimental performance, we conducted the experiments separately for the samples with and without the removal of baseline data and the average results of the multiple experiments are shown in Table 3. ALL in the experimental data refers to the set of physiological signals containing BP, HR, RR, PR, SpO_2_, and SC.

The article "The Method for Identifying Employees' Emotions in Adverse States Incorporating PSO-kNN Algorithm and Multiple Physiological Parameters" was published in 2022. Journal: Comput Intell Neurosci.

The effect of the comparison of the average recognition rate of the un-baselined versus the baselined in the recognition results of the three types of emotional states and the three levels of tension in the adverse state is shown in Figure 3.

In order to identify the level of tension in poor states, 30 samples were drawn from a dataset of 42 tension level samples for training and the remaining 12 were used for testing. In order to conduct sufficient experiments to test the recognition effect in multiple situations, multiple experiments were conducted in both situations and the average of the multiple experiments was used as the final result. We conducted separate experiments on samples with and without the removal of baseline data, and the recognition results for the test set are shown in Table 4.

A comparison of the number of features of the optimal subset for the two cases is shown in Figure 4.

Particle swarm optimisation algorithms allow collaboration and information sharing between individuals in a population to find the optimal solution, which has the advantage of being simple and easy to implement and does not require many parameters to be adjusted. The results of kNN and PSO-kNN with the removal of baseline physiological data are presented in Table 5

A visual comparison of the recognition rates between kNN and PSO-kNN with the removal of baseline physiological data is shown in Figure 5.

The results of the kNN and PSO-kNN without the removal of baseline physiological data are shown in Table 6.

A visual comparison of the recognition rates between kNN and PSO-kNN without the removal of baseline physiological data is shown in Figure 6.

The IAPS picture system was used in the study here to design the emotion arousal experiment, which was evaluated using a subject emotion arousal questionnaire with high reliability. It can be concluded from the data in Tables 3 and 4 that when using the PSO-kNN algorithm for the identification of adverse emotions, the average recognition rates for all three different emotions were lower than the average recognition rates for the three different levels of tension and that the data processing results without the removal of the baseline data were lower than the recognition results with the removal of the baseline physiological signal. This indicates that the removal of the baseline physiological signals can effectively improve the recognition of emotions in adverse states by eliminating the differences in physiological signals between individuals. Another very important finding is that the selected combination of signals is more accurate than the single signal feature.

The article "The Method for Identifying Employees' Emotions in Adverse States Incorporating PSO-kNN Algorithm and Multiple Physiological Parameters" was published in 2022. Journal: Comput Intell Neurosci.

In the training, diastolic blood pressure and heart rate maximum-minimum difference as well as pulse minimum were repeatedly selected as the optimal subset of features for emotion recognition. This indicates that the selected signals play an important role in the recognition of emotions in adverse states. Compared with the recognition results of Nasoz et al. using the kNN algorithm directly, this paper obtained better recognition results by combining the removal of baseline emotions with the PSO algorithm and optimising the selection of multiple features of multiple physiological signals before using kNN classification. Finally, based on the removal of baseline physiological signals, three predictions were made using the kNN-PSO algorithm for each of the three different emotions and three different levels of tension evoked by the experiment, and the predictions obtained are shown in Table 7.

Pie charts of the predicted outcomes for three of these different moods and three different levels of tension are shown in Figure 7.

## 5. Conclusions

In this paper, three types of emotions and three stress levels were induced using IAPS picture visual stimuli and mental calculation task experiments to build up a sample library of emotion-related physiological signals. Six feature vectors for effective recognition of stressful emotions were found through PSO feature optimisation, and the kNN algorithm was used to achieve emotion calculation and stress level recognition under adverse states. Experimental results show that the PSO-kNN algorithm achieves an effective recognition rate of 75% for the three emotions and 83.33% for the stress level. Through baseline data removal and PSO feature optimisation, the recognition results are better compared to the traditional kNN without feature optimisation selection. It provides some reference for the research of physiological signal processing and pattern recognition algorithms in affective computing research. Due to the limited sample data at present, it is difficult to test the deeper performance of the model. Future work will further expand the sample of emotion-related data in bad states, study the model with better performance for emotion recognition algorithm, and make the model work faster by considering the weighting relationship of the parameters in the PSO and kNN algorithms in more samples. Finally, we aim to extend the emotion recognition model to practical applications to make a real contribution to social change.

## Figures and Tables

**Figure 1:** Visual comparison of the effect value and arousal of four different emotion-evoking picture materials.

The article "The Method for Identifying Employees' Emotions in Adverse States Incorporating PSO-kNN Algorithm and Multiple Physiological Parameters" was published in 2022. Journal: Comput Intell Neurosci.

**Figure 2:** Structure of the specific distribution of features extracted from the six physiological signals.

**Figure 3:** Comparison of the identification results of the (a) three types of emotional states and (b) three levels of tension.

**Figure 4:** Comparison of the number of features of the optimal subset for the two types of cases: (a) three types of emotional states and (b) three levels of tension.

**Figure 5:** Visual comparison of recognition rates between kNN and PSO-kNN with the removal of baseline physiological data.

**Figure 6:** Visual comparison of kNN and PSO-kNN recognition rates without removal of baseline physiological data.

**Figure 7:** Pie charts of predicted outcomes for (a) three different emotions and (b) three different levels of tension.

**Table 1:** Efficacy values and arousal levels of the four IAPS emotion-evoking picture materials.

Emotions	Image RMS	Image wakefulness
Excitement	6.0 ± 0.5	6.5 ± 0.5
Boredom	3.0 ± 0.5	3.5 ± 0.5
Fear	2.0 ± 0.5	7.0 ± 0.5
Calm	5.0 ± 0.5	4.0 ± 0.5

**Table 2:** Characteristics of the six physiological signals extracted.

Physiological signals	Extraction characteristics
Blood pressure	Systolic, diastolic, and systolic-diastolic differential

Heart rate, respiratory rate, pulse rate, oxygen saturation, and skin impedance	Mean, variance, first-order difference mean, maximum, minimum, maximum-minimum difference

**Table 3:** The classification of three stress emotions by physiological signals and their features' combination.

Physiological signals	Number of original features	Optimal subset feature number		Average recognition rate (%)	
		Not to baseline kNN	Removal of baseline kNN	Not to baseline kNN	Removal of baseline kNN
BP	3	2	1	41.67	50.00
HR	6	2	2	50.00	66.67
RR	6	3	3	58.33	66.67
PR	6	2	3	58.33	66.67
SpO_2_	6	1	1	33.33	33.33
SC	6	2	1	58.33	66.67
ALL	33	7	7	66.67	75.00

**Table 4:** The classification of three tension degrees by physiological signals and their features' combination.

Physiological signals	Number of original features	Optimal subset feature number		Average recognition rate (%)	
		Not to baseline kNN	Go to baseline kNN	Not to baseline kNN	Go to baseline kNN
BP	3	1	2	33.33	41.67
HR	6	3	2	58.33	66.67
RR	6	2	1	58.33	58.33
PR	6	3	2	50.00	58.33
SpO_2_	6	1	1	33.33	33.33
SC	6	3	2	50.00	66.67
ALL	33	6	5	75.00	83.33

**Table 5:** Recognition rate results of kNN and PSO-kNN with the removal of baseline physiological data.

Category	Average recognition rate (%)	
	kNN	PSO-kNN
BP	50.00	66.67
HR	66.67	75.00
RR	66.67	66.67
PR	66.67	75.00
SpO_2_	33.33	50.00
SC	66.67	75.00
ALL	75.00	83.33

**Table 6:** Recognition rate results between kNN and PSO-kNN without removal of baseline physiological data.

Category	Average recognition rate (%)	
	kNN	PSO-kNN
BP	33.33	50.00
HR	58.33	75.00
RR	58.33	75.00
PR	50.00	66.67
SpO_2_	33.33	58.33
SC	50.00	75.00
ALL	75.00	83.33

The article "The Method for Identifying Employees' Emotions in Adverse States Incorporating PSO-kNN Algorithm and Multiple Physiological Parameters" was published in 2022. Journal: Comput Intell Neurosci.

**Table 7:** Three sets of emotion-evoking experiments with three different emotions and three different levels of tension.

Experimental group	Accuracy (%)	
	Three stress emotions	Three tension degrees
1	75.00	83.33
2	83.33	91.67
3	83.33	91.67

## Data Availability

The data used to support the findings of this study are available from the corresponding author upon request.
